# Applications of Functionalized Hydrogels in the Regeneration of the Intervertebral Disc

**DOI:** 10.1155/2021/2818624

**Published:** 2021-08-19

**Authors:** Caiping Yan, Xingkuan Wang, Chao Xiang, Yong Wang, Chaoyu Pu, Lu Chen, Ke Jiang, Yuling Li

**Affiliations:** Department of Orthopaedics, Affiliated Hospital of North Sichuan Medical College, No. 1 The South of Maoyuan Road, Nanchong, Sichuan 637000, China

## Abstract

Intervertebral disc degeneration (IDD) is caused by genetics, aging, and environmental factors and is one of the leading causes of low back pain. The treatment of IDD presents many challenges. Hydrogels are biomaterials that possess properties similar to those of the natural extracellular matrix and have significant potential in the field of regenerative medicine. Hydrogels with various functional qualities have recently been used to repair and regenerate diseased intervertebral discs. Here, we review the mechanisms of intervertebral disc homeostasis and degeneration and then discuss the applications of hydrogel-mediated repair and intervertebral disc regeneration. The classification of artificial hydrogels and natural hydrogels is then briefly introduced, followed by an update on the development of functional hydrogels, which include noncellular therapeutic hydrogels, cellular therapeutic hydrogel scaffolds, responsive hydrogels, and multifunctional hydrogels. The challenges faced and future developments of the hydrogels used in IDD are discussed as they further promote their clinical translation.

## 1. Introduction

Low back pain is a leading cause of musculoskeletal disability and places a heavy burden on global healthcare systems. More than 632 million people are affected by low back pain, and its incidence is increasing as the world population ages [1, 2]. Intervertebral disc degeneration (IDD) is one of the leading causes of low back pain. The main treatment modalities for IDD are conservative and surgical, which include anti-inflammatory analgesia, physical therapy, epidural injections, surgical decompression, disc replacement, and vertebral fusion [3]. While conservative treatment cannot prevent the progression of IDD, patients treated surgically are exposed to the risk of surgical complications, postoperative symptom recurrence, and adjacent segment degeneration [4]. Due to the limitations of these conventional therapies, alternative treatments such as cytokine therapy, stem cell therapy, gene therapy, and tissue engineering have been proposed [5–7]. These treatments have been used primarily in animal experiments, although the rare clinical use of these therapies has yielded satisfactory results.

Hydrogels are widely used in biomedical engineering. As hydrogels have similar mechanical characteristics to nucleus pulposus tissue, the use of hydrogels in the treatment of IDD has been a hot topic of recent research [8]. Hydrogels are three-dimensional hydrophilic polymers with a high water content and biocompatibility. They are similar to the natural extracellular matrix (ECM) and can be used as carriers for the delivery of drugs, proteins, and stem cells [9]. As early as the mid-1990s, Raymedica developed a nucleus pulposus prosthesis using polyacrylonitrile-polyacrylamide copolymer and polyethylene fiber that was used in clinical practice. The Aqarelle and BioSic prostheses, injectable protein hydrogels for nucleus pulposus replacement, were developed [10–12]. However, these hydrogel prostheses could only be used to replace the nucleus pulposus and were unable to promote the regeneration and repair of the nucleus pulposus tissue. Moreover, they carried a risk of injury from the implantation process and due to prosthesis displacement, limiting their application [13]. With the development of biomaterial engineering, newly developed multifunctional hydrogels have a broader use in IDD regeneration.

In this review, we discuss the development of multifunctional hydrogels for IDD and regeneration: (1) we introduce the concepts of homeostasis and degeneration of the intervertebral disc and the types of hydrogels used in the treatment of IDD; (2) we classify and summarize the advantages of multifunctional hydrogels in IDD and regeneration; (3) we emphasize the principles behind the use of hydrogels in the treatment of IDD and the high standards of regenerative medicine by customizing their functions. This review is aimed at introducing the biomedical potential of hydrogels, in particular their unique regenerative function in the treatment of IDD, and at providing guidance for the further development of multifunctional hydrogels.

## 2. Homeostasis and Degeneration of the Intervertebral Disc (IVD)

### 2.1. IVD Homeostasis

The normal human spine contains a total of 23 intervertebral discs. The IVD anatomically consists of three parts: the nucleus pulposus, annulus fibrosus, and cartilaginous endplate [14]. The IVD is the largest avascular tissue in the body, with only a few blood vessels and nerves located on the outside of the annulus fibrosus. The IVD is primarily composed of a large amount of ECM, with scattered IVD cells within it. The ECM of the IVD is primarily composed of collagen, proteoglycans, mucopolysaccharides, hyaluronic acid, and a variety of other proteins (such as actin, fibromodulin, and cartilage oligomeric matrix protein) [15]. Type I and type II collagen account for more than 80% of the total ECM of the IVD [16]. IVD cells account for only about 1% of the IVD volume [17], and they play an essential role in the synthesis and secretion of the ECM and the maintenance of the physiologic homeostasis of the IVD.

There are several crucial physiologic homeostasis states in the normal IVD: immune homeostasis, cellular homeostasis, ECM homeostasis, and nutritional homeostasis. The maintenance of these balances is essential to the normal physiologic function of the IVD. The various forms of IVD homeostasis are closely related and maintain a dynamic physiologic balance that changes as the host ages: (1) immune homeostasis means that immune cells are not found in the IVD under normal circumstances due to the annulus fibrosus, cartilage endplates and the protection of FasL and other molecular mechanisms; (2) cellular homeostasis plays a central role in the maintenance of IVD physiology. IVD cells maintain the normal physiologic functions of the IVD by synthesizing and secreting ECM-related proteins; (3) as the main component of the IVD, the ECM bears its biological stress and provides a mechanical scaffold and nutritional supply for IVD cell survival, thereby playing a vital role in cell growth, proliferation, metabolism, migration, and adhesion; (4) nutritional homeostasis is necessary to ensure the normal physiologic function of the IVD. The IVD is an avascular tissue. Essential nutrients such as glucose, oxygen, and the precursors for ECM synthesis are transported around the IVD by the blood and spread throughout the IVD through osmosis; (5) oxygen homeostasis is an integral part of nutritional homeostasis. Neither hypoxia nor normoxia is the most suitable living environment for IVD cells.

### 2.2. Degeneration and Microenvironment Changes

When homeostasis is disrupted by internal or external factors such as genetics, stress, aging, infection, metabolic abnormalities, and smoking, the IDD process begins. The start of this process is largely asymptomatic. The pathologic development of IDD will also accelerate the imbalance in IVD homeostasis. Most of the research on the mechanisms behind IDD focuses on the core of its steady-state imbalance. Internal and external factors that lead to the disruption of IVD homeostasis include: (1) genetic factors. Genetic diversity studies can explain the susceptibility of certain populations to IDD [18, 19]. Recent studies have found that long noncoding RNA can accelerate IDD by affecting the apoptosis of IVD cells and the synthesis of related proteins. Wan et al. [20] performed KEGG analysis on these RNAs and found that the upregulated expression of RP11-296A18.3 could improve FAF1-mediated apoptosis, suggesting that microRNAs and long noncoding RNA play an important role in IDD; (2) biomechanical changes are important external disruptors of IVD homeostasis. In order to maintain an upright position and upper limb movement, the human disc is subjected to significant biologic forces. These stimuli can affect the metabolism and function of the cells of the disc. A certain amount and direction of physical forces encourages disc cells to maintain a normal physiologic state [21, 22]. However, overloaded physiologic stress on the IVD can lead to IDD through the imbalance of multiple homeostasis factors within the IVD. Noguchi et al. [23] found in an animal study that repeated high-intensity loading could lead to the destruction of the medial annulus fibrosus and the instability of the anatomic structure of the IVD. By studying a new mechanical model of the animal spine, Berger-Roscher et al. [24] found that complex stress stimulation could lead to structural destruction of the cartilage endplate and the annulus fibrous. High-pressure culture can induce increased expression of IL-1*β* and IL-6 by nucleus pulposus cells [25], and the high expression of these inflammatory cytokines has a potentially adverse effect on IVD immune homeostasis. Nonphysiologic stress can induce nucleus pulposus cell apoptosis and disrupt intercellular interstitial osmosis, thereby interrupting IVD nutrient homeostasis and oxygen homeostasis; (3) aging also impacts IVD homeostasis. IDD is present in approximately 40% of people under 30 years old [26] and more than 90% of people over 50 years old [27]. As the human body grows older, IVD homeostasis gradually becomes unbalanced and damaged. Various pathologic changes such as the accumulation of inflammatory mediators, the formation of cell clusters, nucleus pulposus fibrosis, annulus fibrosus rupture, and cartilaginous endplate calcification can be observed in the aging IVD [28]. The ability of aging disc cells to secrete ECM-associated proteins is significantly reduced, affecting ECM homeostasis. At the same time, the normal physiologic structures of the annulus fibrosus and the cartilage endplate in the aging IVD are destroyed, which results in antigen exposure. Decreased FasL expression by the aging nucleus pulposus cells reduces the active elimination of infiltrating immune cells at the molecular level [29]. These changes may lead to imbalanced IVD immune homeostasis. Further calcification of the cartilaginous endplate caused by aging can be a barrier to nutrient penetration, thereby disrupting the nutrient and oxygen homeostasis of the IVD and accelerating IDD [30]. However, some pathologic changes may not directly be related to aging, which is indicative of the complexity of the IDD disease course; (4) in addition to the above factors, additional pathologies such as infection, diabetes, and smoking may contribute to IDD [31].

In summary, IDD is a complex process that involves genetics, the environment, and cellular senescence. Understanding the mechanisms behind IDD is necessary to appropriately design biomaterials for the treatment of IDD. Hydrogels, which are analogs of the ECM, provide structural support for the regeneration of nucleus pulposus cells, guide the differentiation of nucleus pulposus cells and the production of ECM, and act as a carrier of drugs or stem cells, and are therefore lead candidate materials for the treatment of IDD.

## 3. Types of Hydrogels

### 3.1. Synthetic Hydrogels

Synthetic hydrogels are three-dimensional network microstructures that are formed by the combination of hydrophilic molecules and synthesized by hydrogen bonds or covalent bonds followed by complete hydration and swelling. Synthetic hydrogels include polyacrylic acid, polyacrylic acid salts, polyacrylamide derivatives, polyvinyl oxide, derivative copolymers, polyvinyl alcohol, polyphosphazene, and polypeptides. Although synthetic hydrogels can overcome the shortcomings of the insufficient mechanical properties of natural hydrogels, they also have limitations that include the need to add toxic components during the preparation process, their slow degradation, and their insufficient biologic activity. Synthetic hydrogels are therefore rarely used alone in tissue engineering and are used instead to augment natural hydrogels.

Polyvinyl alcohol (PVA) is a hydrogel that has stable chemical properties and biocompatibility. Different strategies can adjust its properties [32]. PVA can be created via forge cast drying (CD) and has a morphology, moisture content, and mechanical behavior that is very similar to that of natural cartilage, making it an ideal substitute for articular cartilage [33]. Some PVA-based hydrogel membranes can be used as dressings to promote wound repair and antimicrobial effects [34]. PVA cryogel has similar mechanical properties to the human IVD, a high water content, and good biocompatibility, making it a promising new tissue biomimetic IVD material [32].

Polyethylene glycol (PEG) is a hydrophilic polymer. Hydrogels based on PEG are widely used in various biomedical fields because of their easy synthesis and tissue-like properties [35]. Peptide- and protein-functionalized PEG norbornene hydrogels were prepared by combining thio-transforming growth factor *β*1 with PEG hydrogel and cross-linking it with an MMP-degradable polypeptide. This hydrogel can be cleaved by enzymes present in the surrounding tissues in a short period of time, thus promoting cartilage matrix formation [36]. Laminin 111 (LM111) was the first polyethylene glycosylated with acrylic-PEG-NHS (AC-PEG-NHS). A PEG-LM111 conjugate was mixed with PEG-DA and cross-linked using ultraviolet light to form a PEG-LM111 hydrogel. The LM111-functionalized PEG hydrogel promoted the aggregation, differentiation, and production of glycosaminoglycan (GAG) in primary nucleus pulposus cells in a 3D cell culture model [37]. Frith et al. [38] reported that a PEG/HA hydrogel prepared by cross-linking 3-4-hydroxyphenylpropionic acid-functionalized PEG with tyramine-functionalized hyaluronic acid had properties that were suitable for nucleus pulposus regeneration. Moreover, this work confirmed that covalently linking pentosan polysulfate (PPS) to HA maintained PPS's bioactivity and had excellent chondrogenic capacity.

Poly(lactic-co-glycolic) acid (PLGA) is an aliphatic polyester copolymer that has good biocompatibility and biodegradability [39, 40]. It is versatile, easy to modify, and approved by the Food and Drug Administration and the European Medicines Agency for various clinical applications. PLGA is often used as a carrier for drug or stem cell delivery using microspheres, nanoparticles, and nanofibers to improve drug solubility, efficacy, effectiveness, and safety [41]. We have previously designed a medical robotic microsphere attached to PLGA to carry human adipose mesenchymal stem cells *in vitro* to target a cartilage defect via magnetism [42]. Zhang et al. [43] injected simvastatin-loaded poly(ethylene glycol)-poly(lactic acid-co-glycolic acid)-poly(ethylene glycol) hydrogel in a rat model of IDD. The hydrogel's dual effect of promoting autologous chondrogenic disc repair and delaying disc degeneration may provide an inexpensive and easy-to-use treatment strategy for IVD regeneration.

### 3.2. Natural Hydrogels

Natural hydrogels are usually derived from animal and plant extracts; many of which are essential components of human tissues and organs. Natural hydrogels are nontoxic, have a high degree of biologic safety, and possess a high level of biocompatibility. Natural hydrogels, owing to their significant biocompatibility, are widely used in tissue regeneration and repair. Commonly used natural hydrogels include gelatin, collagen, fibrin, hyaluronate, alginate, agarose, and chitosan. Biomaterials based on natural hydrogels for bone tissue engineering applications have begun to be translated into the clinic [44, 45].

Hyaluronic acid (HA), a linear polysaccharide macromolecule, is an essential component of the ECM of cartilage. It has a high water content and can be degraded by hyaluronidase *in vivo* [46]. HA and its derivatives are often used in tissue engineering and bioengineering to create new biomaterials and have been widely used clinically [47]. Chemically modified HA retains its biocompatibility and biodegradability while providing additional functions [48]. The HA backbone includes several modifiable groups such as its carboxyl group. One of the most extensive modifications of HA is the formation of hyaluronic acid methacryloyl (HAMA) by HA and methacrylic anhydride under alkaline conditions [49]. Chen et al. [50] modified HA with aldehyde and methacrylic acid to create an injectable adhesive hyaluronic acid hydrogel (AHAMA). The aldehyde group of the hydrogel and the amino group of the cartilage tissue were closely bonded to one body through the Schiff base reaction, promoting the combination of new cartilage and natural cartilage and significantly promoting cartilage regeneration.

Gelatin is primarily derived from bovine collagen and porcine collagen through thermal denaturation or lysis [51]. Gelatin contains many MMP and arginine-glycine-aspartic acid sequences, is biodegradable, and promotes cell adhesion *in vivo* [52]. Gelatin has better solubility and lower antigenicity than collagen and can be physically cross-linked into hydrogels at low temperatures. In addition, by introducing methacrylate groups, the gelatin can be photo-cross-linked into a GelMA hydrogel following photoinitiation [53]. Yang et al. [54] prepared GelMA hydrogel microspheres loaded with kartogenin using microfluidics. The GelMA microspheres can repair cartilage defects after delivery via minimally invasive injection via sustained drug release therapy. Similarly, Xu et al. [55] synthesized growth differentiation factor 5-loaded gelatin methacryloyl injectable microspheres (GMs) via electrospraying. GMs were used as adipose stem cell delivery vehicles, exhibited good mechanical properties and biocompatibility, and enhanced the differentiation of the adipose stem cells into a nucleus pulposus cell-like phenotype *in vitro*. GMs can also accelerate ECM synthesis.

Chitosan is the primary derivative of chitin, an amino polysaccharide prepared by the alkaline deacetylation of chitin [56]. It possesses biocompatibility, biologic activity, biodegradation, and significant mechanical strength. Chitosan is also highly soluble, which has expanded its use in the field of biologic materials [57]. Alinejad et al. [58] prepared several novel temperature-sensitive chitosan hydrogels by mixing chitosan with different combinations of sodium bicarbonate (SHC), *β*-glycerophosphate (BGP), and phosphate buffer (PB) and tested the properties of several hydrogels using a rheometer and cell culture. One of the hydrogels (SHC0.075/Bgp0.1) exhibited mechanical properties similar to those of the human IVD, could maintain nucleus pulposus cell activity, and induced a high level of glycosaminoglycan production in the nucleus pulposus cells encapsulated in the hydrogel. The injectable and ECM retention properties of chitosan make it a good hydrogel scaffold for treating early stage IDD [59].

Alginate is a naturally high-molecular-weight polysaccharide that is found in algae and the bacterial cell wall. Sodium alginate is a natural water-soluble polysaccharide block copolymer that is composed of *β*-L-mannoic acid (M) and *α*-L-gulonic acid (G). Sodium alginate can be cross-linked by divalent ions such as calcium [60]. It has many advantageous properties, including biocompatibility, excellent solubility, high porosity, degradability, and adjustable viscosity [61]. Sodium alginate has consequently been used in many biomedical fields such as wound healing, drug delivery, and *in vivo* implantation. Tsujimoto et al. [62] used an absorbable super purified alginate hydrogel to 3D culture human IVD cells and implanted super purified alginate hydrogel into rabbit and sheep discectomy models to simulate postdiscectomy treatment. Their results showed that super purified alginate hydrogel enhanced the activity of human IVD cells and promoted ECM production and has biomechanical properties similar to those of the human IVD. It may therefore be a new treatment strategy for replacing the IVD after a discectomy.

In summary, natural hydrogels and synthetic hydrogels have advantages and disadvantages. Natural hydrogels have good cell affinity because of their specific cell action sites [63], but are not easy to obtain in large quantities and their structure and properties are not easy to adjust. Synthetic hydrogels can be produced on a large scale and adapted to different applications by improving their structure and mechanical properties during the preparation process. However, they lack cell recognition signals and possess poor cell affinity [64].

## 4. The Mechanism and Principles of Hydrogel-Promoted IVD Regeneration

An ideal hydrogel for regenerating the IVD should have the following properties: (1) good biocompatibility and biodegradability; (2) injectability so it can be used as adjuvant therapy for conservative treatment or minimally invasive surgery; (3) in situ curing to avoid leakage; (4) strong biomechanical properties, which improve the differentiation of nucleus pulposus cells; (5) good drug carrying and sustained-release capacity to extend the duration of treatment; (6) can integrate and adhere with the target to prevent poor localization and treatment failure; and (7) can encapsulate stem cells and retain the ECM to promote IVD regeneration.

## 5. Applications of Cell-Free Hydrogels in IVD Regeneration

### 5.1. Applications of Hydrogels Loaded with Traditional Drugs in IVD Regeneration

The inflammatory microenvironment mainly refers to inflammatory cells and inflammatory factors, which are essential pathologic factors in the incidence and development of inflammatory diseases. Inflammatory cytokines play a significant role in the catabolic processes during IDD pathogenesis. Large amounts of matrix metalloproteinases, nitric oxide, prostaglandin E2, IL-1, IL-6, IL-8, and TNF-*α* are overexpressed in the diseased disc. Targeting the inflammatory process is therefore one treatment strategy for treating chronic low back pain and IDD [65]. Traditional COX-2 inhibitors effectively reduce low back pain but also have significant side effects, such as ulcer formation in the digestive tract [66]. Further, because the IVD is avascular, it is often difficult for drugs to reach the treatment site. Hydrogels are widely used as topical anti-inflammatory therapies because they have good drug delivery and controlled release properties [67]. Tellegen et al. [68] used a celecoxib-loaded PCLA-PEG-PCLA injectable hydrogel in a canine model of chronic low back pain caused by IDD. In a 3-month experiment, the hydrogel did not affect the MRI properties of the IVD. A clinical exam and owner questionnaire showed significant back pain improvement in 9 out of the 10 dogs. The inflammatory response time is different in an inflammatory microenvironment. For example, surgical trauma can be inflammatory for more than 14 days, and that inflammation makes disease recurrence highly likely. It is therefore necessary to suppress postoperative inflammation as well [69]. Liu et al. [70] designed an aspirin-loaded hydrogel with similar properties to the ECM to treat local inflammation after a discectomy. The system could be cured in situ at the defect site postoperatively, which is conducive to repairing tissue defects (Figure 1(a)). It also permitted slow drug release. The released anti-inflammatory drugs prevented postoperative inflammatory factor expression. A growing number of studies have shown that multiple factors, such as the macrophage M1/M2, increased reactive oxygen species (ROS) level, and mitochondria-related autophagy, contribute to the chronic inflammation and gradual degeneration of the IVD [71]. Hydrogel-mediated drug delivery may be able to improve this milieu. Bai et al. [72] developed a ROS-scavenging hydrogel scaffold loaded with rapamycin (RapA@Gel), which reduced ROS levels and promoted M2-type macrophage polarization (Figure 1(b)). This represents a new strategy for regulating the local inflammatory microenvironment to promote IVD regeneration.

### 5.2. Applications of Hydrogel Loaded with Growth Factors in IVD Regeneration

Growth factors (GFs) are proteins secreted by cells to stimulate cell proliferation, differentiation, and migration. GFs also regulate ECM metabolism and are responsible for paracrine, secretory, and endocrine function [73]. Tissue fluid in the IVD can transport growth factors through the endplate via an endocrine mechanism because there are no blood vessels. Autocrine and paracrine growth factors are the main regulatory mechanisms of the IVD. Recent studies on the pathogenesis of IDD have shown that GFs are excellent options for treating, reversing, or delaying ID [73]. Research reported that intradiscal injection of osteogenic protein-1 (OP-1) increased disc height 2, 4, and 8 weeks after injection and theorized that OP-1 may act by stimulating metabolic activity. Subsequent biochemical tests showed that the proteoglycan levels in the OP-1 group were higher than those in the saline group 2 weeks after injection. However, there was no difference between the OP-1 group and the saline group at subsequent time points, suggesting that continuous or repeated local GF administration may be required due to their relatively short half-lives [74]. It has also been shown that the direct injection of bone morphogenetic protein 2 (BMP-2) may accelerate the degenerative process [74], and that injection of BMP-2 or OP-1 into the laminectomy or foraminotomy site may result in ectopic ossification and restenosis [75]. There is therefore an urgent need for the development of a continuous drug delivery system to assist with local GF administration in order to reduce side effects and improve treatment efficacy. Platelet-derived growth factor-BB, a major component of platelet-rich plasma, has been effective at various orthopedic applications [76]. Paglia et al. [77] trialed recombinant human platelet-derived growth factor-BB (rhPDGF-BB) added to a HyStem-C thiol-modified hyaluronic acid (TMHA) hydrogel with pEGSSDA in the treatment of IVD in a rabbit model. After eight weeks of treatment, MRI, histologic, and biomechanical tests demonstrated that treatment with rhPDGF-BB preserved the structure and hydration of the degenerative disc. This effect was enhanced when rhPDGF-BB was delivered in the form of a TMHA hydrogel. Henry et al. [78] encapsulated growth differentiation factor-5 (GDF5) and TGF-*β*1 into injectable pullulan polysaccharide microspheres (PMBs) to permit sustained GF release and loaded the microspheres into a self-curing hydrogel composed of silylated hydroxypropyl methylcellulose (Si-HPMC). The system was cross-linked in situ at the disc injury site to achieve disc regeneration. The release time of the GFs from the PMBs was 21 to 28 days. The Young's modulus of the Si-HPMC hydrogel was about 1 kPa, and adding PMBs did not affect the hydrogel's mechanical properties. Injectable hydrogels that deliver cells and/or drugs directly to the nucleus pulposus have attracted great interest over the last decade [79]. These highly hydrated biomaterials can be injected through a small incision, interlaced with tissue defects. They can be designed to mimic the ECM to maintain the activity and function of the nucleus pulposus cells [80]. Hydrogels with shear diluting and recovery properties are therefore of particular interest. Ligorio et al. [80] recently developed an injectable graphene oxide- (GO-) self-assembly peptide FeFKFeFK (F: phenylalanine; K: lysine; E: glutamate) hydrogel (Figure 1(c)). FeFKFEFK (F8) is a very short octapeptide that readily self-assembles into *β*-sheet-rich fibers with a diameter of 3 nm. When critical gel concentration (CGC ~ 5 mg mL^−1^, pH = 4) is exceeded, a self-supporting, transparent, and injectable hydrogel can be formed. The hydrogel adsorbs the growth factors onto the GO sheets and mixes with them (GO/TGF-*β*3 ADS-F8). Subsequent experiments demonstrated that the hydrogels upregulated the expression of the nucleus pulposus markers and produced nucleus pulposus ECM that was rich in collagen. In addition to mechanically enhancing self-assembled peptide hydrogels and providing adhesion sites for cells, GO tablets can also be used as nanocarriers to store and deliver GFs.

### 5.3. Applications of Gene-Carrying Hydrogels in IVD Regeneration

The effectiveness of injectable hydrogels at carrying drugs and/or growth factors to regulate inflammation and cell metabolism at the site of disc degeneration has been demonstrated *in vitro* and *in vivo*. However, these treatments are dose-dependent, and multiple injections may be needed when these impregnated hydrogels are used in larger animals or humans. However, the trauma caused by multiple punctures may counteract the drug's effectiveness and potentially worsen the disc degeneration. Gene therapy, an alternative method for IDD treatment, could potentially alter or reverse the process of IDD by reprogramming the IVD cells [81, 82]. Liang et al. [83] used an adenovirus-mediated human GDF5 gene (Ad-GDF5) to treat a mouse model of IDD. Ad-GDF5 injection promoted chondrocyte proliferation and proteoglycan production and permitted the long-term expression of the target protein in the IVD. The PEO-PPO-PEO copolymer is a nonionic triblock copolymer based on hydrophilic polypropylene oxide (PEO) and hydrophobic polypropylene oxide (PPO) [84]. Madry et al. [85] used this hydrogel to carry a recombinant adeno-associated virus (RAAV) to overexpress the SOX9 transcription factor in full-thickness cartilage defects of miniature pigs. This work illustrates the concept of the use of advanced biomaterials for gene vector delivery, suggesting that cartilage repair via minimally invasive gene delivery is possible and that cartilage repair can occur when the host immune response is disrupted. Several miRNA delivery vectors have been developed for gene therapy, such as viral vectors and liposomes [86]. However, their applications have been limited due to their biotoxicity and immunogenicity [87]. Chen et al. [88] believed that delivering miRNAs to the IVD was a challenge, and that a poor delivery vector could lead to miRNA inactivation, low transfection efficiency, and short half-life. They synthesized a multifunctional PEG hydrogel by cross-linking four-arm SH-PEG with Ag^+^ via Ag-S coordination (Figure 2), which has an excellent agomir load (agomir is a cholesterol-methylated and thiophosphate-modified miRNA fragment that mimics the role of miRNAs in the regulation of target gene expression). This hydrogel system can be injected directly into the intervertebral space through a minimally invasive method and can self-cure in situ after injection, reducing the risk of leakage and rupture. The results suggest that this injectable, self-healing, and biodegradable multifunctional PEG hydrogel can be used as an advanced biomaterial to deliver miRNA874-structured agomir 874 to downregulate the expression of MMPs and normalize the metabolic balance of the ECM in the nucleus pulposus to slow the progression of disc degeneration. Moreover, this “gene-hydrogel” microenvironment can also be applied to the treatment of other diseases, expanding the applications of gene therapy.

## 6. Applications of Hydrogel/Cell Therapy in the Regeneration of the IVD

The initial signs of IDD occur in the nucleus pulposus and include decreased cell density, reduced water content, and the loss of the ECM and proteoglycans. Reducing the number and function of the nucleus pulposus cells is one of the most critical parts of IDD, and restoration of the deformed nucleus pulposus is key to its treatment [89]. Cell-based therapeutic strategies in animal studies of IDD have shown that mesenchymal stem cells (MSCs) injected into the nucleus pulposus can survive for several months and induce ECM production. Orozco et al. [90] performed a pilot study on the feasibility and safety of MSCs in patients with chronic degenerative disc disease, showing that cell-based alternative therapy is simpler, less invasive, and safer than conventional therapy. More recent works have employed biomaterials with cell-protective effects to protect stem cell activity. Hydrogels with biocompatibility and injectable properties have aroused the greatest interest. As a supportive scaffold, hydrogels can improve cell survival and mimic their natural environment. Considering that restoration of disc height may be key to tissue regeneration, Richardson et al. [91] inserted hMSCs into a chitosan-glycerol phosphate (C/GP) gel and cultured them in standard medium for 4 weeks. The authors found that the MSCs expressed chondrocyte phenotypes but did not express osteogenic marker genes or cell hypertrophy markers. Moreover, the chondrocyte gene marker expression of the MSCs was similar to that of nucleus pulposus cells and articular chondrocytes. However, the degree of synthesis and deposition of ECM proteins by the MSCs in the gel was higher, and the degree of MSCs matching with nucleus pulposus cells was higher than that of articular chondrocytes. This demonstrated that C/GP hydrogels impregnated with MSCs may provide a minimally invasive and clinically feasible treatment for IDD. Furthermore, Clark et al. [92] found that integrin-specific hydrogels can regulate hMSC adhesion, paracrine signal, and osteoblast differentiation in mouse bone defects. This hydrogel promotes tissue healing by promoting the survival and repair activities of hMSC.

Alginate brine hydrogels are often used to encase BMSCs in order to induce cartilage or nucleus pulposus cell formation [93]. Zeng et al. [94] suggested that alginate brine hydrogels usually require *in vitro* polymerization before *in vivo* implantation (Figure 3), thus impairing their injectable properties in restricted and high-pressure nucleus pulposus environments. Polyethylene glycol-diacrylate microcrystalline glass (PMS) was used as the skeleton network of the alginate brine gel. Sodium alginate precursors and BMSCs were loaded into PMS and then polymerized. The compression modulus of the PMS loaded with sodium alginate was similar to that of the nucleus pulposus. *In vitro* experiments verified that PMS loaded with sodium alginate can be easily injected into the canine IVD through a small-caliber needle, and that treatment reduced nucleus pulposus degeneration through a minimally invasive, low cell damage treatment.

Laminin, a derivative of the ECM, can regulate the morphology of nucleus pulposus cells and promote the differentiation of the immature nucleus pulposus [95]. Francisco et al. [96] developed an injectable laminin-functionalized PEG hydrogel with tunable mechanical properties that could be used as a biomaterial for transporting cells to the IVD. Although stem cell therapy has potential, direct injection of stem cells into the nucleus pulposus may lead to osteophyte formation, which can exacerbate disc degeneration [97]. Chen et al. [98] cultured adipose stromal cells (ASCs) in a light cross-linked gelatin-methacrylate hyaluronic acid hydrogel (GELHA). The hydrogel effectively promoted the transformation of the integrin *β*v*α*6 into activated transforming growth factor 1, which promotes the nucleus pulposus-like differentiation of ASCs and ECM synthesis. Furthermore, it was verified in a rat IVD model that the combination of this hydrogel and ASCs could significantly improve the efficacy of ASCs in IVD repair.

At present, the 3D bionic hydrogel scaffold based on bioprinting has made a significant breakthrough in treating spinal cord injury [99]. We believe that the future novel hydrogel can also make significant achievements in IDD treatment, including the ability to withstand physiologic pressures, support the biologic activity of MSCs, and have a high enough porosity to permit the diffusion of growth factors, oxygen, and nutrients in order to effectively induce cartilage and nucleus pulposus cell regeneration.

## 7. Applications of Responsive Hydrogels in IVD Regeneration

### 7.1. Applications of Temperature-Responsive Hydrogels in IVD Regeneration

Temperature-responsive hydrogels usually contain hydrophilic and hydrophobic groups and can undergo phase transformation at a specific temperature, thereby permitting hydrogel morphology to change with swelling. This temperature is known as the minimum critical solution temperature (LCST) or the maximum critical solution temperature (UCST) [100]. Temperature-responsive hydrogels used to prepare intelligent drug delivery systems are typically hydrogels with LCST. When the environmental temperature is lower than the hydrogel's LCST, the hydrophobic effects between its polymer chains are weak and the hydrogel enters a hydrophilic swelling state. This state makes the hydrogel injectable. In contrast, when the temperature of the hydrogel is at or above its LCST, the hydrophobic interactions between the hydrogel's polymer chains increase significantly and the hydrogel contracts into a dense networked structure. A typical example of a temperature-responsive hydrogel is the PEG and polypropylene glycol copolymer (PPG) with LCST or the PEG-PPG-PEG triblock copolymer. The network formation of this kind of hydrogel depends on the self-assembly of the hydrophobic PPG and the hydrophilic PEG. When its temperature rises to LCST, the polymer changes from solid to gel [101, 102]. The LCST of this hydrogel can be adjusted by the length of the PEG and PPG chains. A newer generation of PLGA-PEG-PLGA triblock copolymer hydrogels has recently been developed that undergoes a solid-gel-solid transformation that is regulated by the length of the chain segment [103, 104]. Compared with PEG-PLGA-PEG, PLGA-PEG-PLGA is significantly less difficult to synthesize and has a lower critical gel concentration and temperature transition point.

Recent works have used temperature-responsive hydrogels in the treatment of IDD. Li et al. [105] successfully synthesized a thermally sensitive N-hexanol chitosan (HGC) hydrogel and used it as a minimally invasive injectable treatment of disc herniations in rabbits. This hydrogel has a heat-sensitive solid-gel transition (25~56°C) and exhibits long-term stability. The biocompatibility of the HGC hydrogel was also demonstrated in a pig IDD model. Pan et al. [106] prepared a thermal hydrogel that delivered a controlled release of gefitinib to treat IDD. This hydrogel not only inhibited ECM degradation but also promoted type II collagen synthesis. These results suggest that the heat-sensitive injectable HGC hydrogel may be a potential nonsurgical treatment of IDD. Although temperature-responsive hydrogels exhibit form-changing properties within a physiologic temperature range, the complexity of their preparation process, the need for many organic reagents, and their irreversible gelation mechanism limit their practical applications in the biomedical field. Further research is therefore necessary.

### 7.2. Applications of Enzyme-Responsive Hydrogels in IVD Regeneration

In addition to temperature-responsive hydrogels, another vital type of chemically responsive hydrogel is the enzyme-responsive hydrogel. Enzyme-responsive hydrogels are generally composed of enzyme-responsive polypeptides that can change their configuration or break when catalyzed by specific enzymes. The degradation products of polypeptide hydrogels are all amino acids, which generally do not cause a nonspecific immune reaction in the human body. These polypeptides and their derivatives have therefore been studied extensively as components of enzyme-responsive hydrogels. The most widely studied enzyme-responsive hydrogels include glutamine transaminase-responsive hydrogels, kinase/phosphatase-responsive hydrogels, tyrosinase-responsive hydrogels, peroxidase-responsive hydrogels, esterase, and endonuclease-responsive hydrogels.

The use of enzyme-responsive hydrogels in IDD and repair has partially been reported. Zheng et al. [107] developed a H_2_S-releasing hydrogel system with both a pH and enzymes capable of treating IDD. This hydrogel is fairly stable under neutral conditions; however, in the acidic pH and high MMP levels of the IDD environment, the hydrogel loses its cross-linked state, resulting in the rapid release of H_2_S. This makes this hydrogel a potential treatment option for IDD. Feng et al. [108] developed an injectable MMP-cleavable hydrogel to encapsulate the MMP-responsive miR-29a multimicelle system (Figure 4). The system first triggers hydrogel degradation by sensing an increase in local MMP level, thereby targeting the degenerated IVD tissue and releasing multimicelles. The release of the multimicelles in response to the MMP detaches the PEG shell and is followed by enhanced cellular uptake and endosomal escape from the nucleus pulposus cells. This system respects that the efficient transmission of miRNA can continuously inhibit MMP-2, which provides a new universal method for local gene therapy in the setting of chronic disease. In addition, Frith et al. [109] produced an enzyme cross-linked polyethylene glycol/hyaluronic acid hydrogel scaffold system that demonstrated good immune tolerance when injected subcutaneously in rats and could induce chondrogenesis of mesenchymal precursor cells, which supported its obvious potential as a tissue engineering material. It also provided a new idea for the treatment of IDD.

Enzyme-responsive hydrogels have many advantages, such as adjustable degradation time and controllable cell behavior, and have potential as carriers that can permit controlled and sustained drug release. The design of reasonable self-assembled hydrogels that use mild and biocompatible enzymatic cross-linking methods to regulate their strength and demonstrate improved cell recognition activity and biodegradability will bring more solutions to the field.

### 7.3. Applications of Other Stimulus-Responsive Hydrogels in IVD Regeneration

Stimulus-responsive hydrogels also include pH-responsive hydrogels, glucose-responsive hydrogels, magnetic responsive hydrogels, and light-responsive hydrogels [110]. Stimulus-responsive hydrogels have recently undergone rapid development in the field of tissue engineering. However, they still have a long way to go before they can be used clinically. For example, the effects of the properties of the hydrogel and the structure of the tissue engineering scaffolds on the target cells are not completely understood, and the construction of bioactive tissues with complex vascular systems is still a significant problem. The development of new hydrogels with good bioactivity and safety for the human body remains a significant challenge.

## 8. Applications of Multifunctional Hydrogels in IVD Regeneration

### 8.1. Applications of Interpenetrating Network Hydrogels (IPN) in IVD Regeneration

Hydrogels are usually formed from biopolymers via chemical cross-linking or molecular interactions. They possess many of the advantages of biopolymers, such as bioactivity, biocompatibility, and degradability. However, these hydrogels generally have weak mechanical properties [111]. Song et al. [112] suggested that modifying histones by mechanical cues (including matrix stiffness, mechanical stretch, and shear stress) to modulate stem cell differentiation and cell reprogramming can facilitate epigenetic changes in cell phenotypic transformation. For this reason, some researchers increased biopolymer concentrations or cross-linking densities to improve the hydrogel's mechanical properties, but these methods can negatively affect the activity of the loaded cells by impeding the diffusion of growth factors, nutrients, and other substances. The potential of hydrogels with poor mechanical properties in the regeneration of the IVD is therefore limited. In order to improve the performance and bioactivity of biopolymer hydrogels, IPN hydrogels have been designed. IPN hydrogels are hydrogels with interconnected networks of two or more independent biopolymers cross-linked in a synchronous or sequential chemical/physical manner [113]. Compared with traditional hydrogels, IPN hydrogels have increased controllability, better mechanical strength, and can accept a high degree of drug loading [114]. Gullbrand et al. [115] believed that the nucleus pulposus would be subjected to higher compression strains during the late stages of IDD. The hydrogel's mechanical properties were therefore considered critical. However, the mechanical properties of most applied hydrogels are inadequate, leading to their collapse during long-term compression and their inability to support the regeneration of the nucleus pulposus over space and time. An IPN hydrogel consisting of an oxidized glucan, amino-modified gelatin, and a 4-arm polyethylene glycol-acrylate (4APEG-ACR) was therefore developed. This IPN hydrogel has good cell compatibility and injectability and can exhibit enhance toughness by adjusting the proportion of its hydrogel network. Injection of IPN hydrogel into a nucleus pulposus defect in animal models promoted regeneration of the IVD. Moffat et al. [116] developed a hydrogel that consisted of a triple IPN of dextran, chitosan, and sclerostin, which they then injected into the degenerated lumbar IVD of goats. The authors showed that the hydrogel could support the activity of the nucleus pulposus cells and MSCs, possessed the ability to produce ECM *in vitro*, and could effectively regenerate the degenerative goat lumbar IVD *in vivo*. Caliari and Burdick [117] developed a MSC seed fiber composite by soaking MSC-coated agarose hydrogels in PEG-DA and then cross-linking them to form IPN hydrogels (Figure 5(a)). The hydrogels were then permeated into 3D woven PCL scaffolds, thereby showing that the hydrogel system has biomimetic mechanical properties and supports the survival and differentiation of MSCs, which provides a new direction for IVD regeneration.

### 8.2. Applications of Hydrogel Microspheres in IVD Regeneration

Hydrogels have generally been used as drug delivery carriers and substrates for cell culture. Hydrogels are traditionally cross-linked into blocks with nanoscale network voids inside, permitting the spread of multiple molecules [117]. However, block hydrogels are often limited by their large size, especially when they need to be injected into the IVD. New methods such as batch emulsions, lithography, electrohydrodynamic spraying, mechanical fragmentation, and microfluidic emulsions have been developed as alternative strategies for hydrogel microsphere preparation [118]. Compared with traditional block hydrogels, hydrogel microspheres retain the original characteristics of the hydrogel and have a larger specific surface area. Moreover, they can be injected through tiny needles. Hydrogel microspheres can exist independently of each other or cluster together to perform different functions. Bian et al. [119] prepared GelMA hydrogel microspheres using microfluidic technology. After surface modification of the microsphere, the active peptide APETX2 was covalently coupled to it. The microsphere was then used to load nucleus pulposus cells to form an injectable “peptide-cell-hydrogel” microsphere (Figure 5(b)). *In vivo* and *in vitro* experiments verified that this new hydrogel microsphere system could effectively reduce the production of inflammatory factors and promote ECM deposition by the loaded nucleus pulposus cells in a rat model of IDD. Hodgkinson et al. [120] designed an injectable PLGA/PLGA-PEG-PLGA microsphere loaded with rhGDF6, which has a high encapsulation rate of growth factors and controlled release. The microsphere system sustained the release of rhGDF6 for 14 days *in vitro*. This system also induced ASC differentiation into the nucleus pulposus cells and produced nucleus pulposus-like ECM that was rich in acrasin.

### 8.3. Applications of Self-Assembled Nanopolypeptide Fiber Hydrogels in IVD Regeneration

Self-assembled nanopolypeptide hydrogels are a new member of the hydrogel family. As a new molecular engineering scaffold material, self-assembled nanopolypeptide hydrogels have been widely studied for their roles in regenerative medicine, 3D cell culture, and sustained drug release. Self-assembled nanopolypeptide hydrogels have been used to repair cartilage [121] and dental pulp [122]. They exhibit the following characteristics: (1) their nanofibers are synthesized from natural amino acids, avoiding the contamination of foreign proteins (such as collagen scaffolds, matrix adhesive, and laminin) [123]; (2) their nanofibers can quickly self-assemble into a hydrogel of nanofibers similar to the structure of ECM *in vivo*, with a water content as high as 99%; (3) their degradation products exhibit good biocompatibility; (4) their nanofibers should have good biologic activity, which is beneficial to the adhesion, growth, proliferation, differentiation, and matrix synthesis of the seeded cells; (5) their nanofibers can be injected into the body through a minimally invasive method; (6) their nanofibers can guide tissue regeneration. These factors make self-assembled polypeptide nanofiber hydrogels very promising materials for the regeneration of the nucleus pulposus.

The discovery of self-assembled nanopolypeptide fiber hydrogels provides a new opportunity for IVD regeneration. Novel functionalized self-assembled polypeptide nanofiber hydrogels can be constructed by connecting short functional fragments with biologically active components at the C-terminal of Rada16-I [124]. Chao-Feng et al. [125] confirmed that BMP-7 exhibits superior IVD regenerative function in an animal model. However, the short half-life and limited action time of BMP-7 limit its clinical applications. Chen and Webster [126] found that SNVI, KPSS, and KAIS3 short active fragments exhibited critical biologic activities similar to those of BMP-7. It was therefore possible to prolong the half-life of BMP-7 by combining it with the C-terminal of the self-assembled polypeptide Rada16-I. Tao et al. [127] applied this functionalized self-assembled polypeptide hydrogel to regenerate degenerated human nucleus pulposus cells with good effect. Wu et al. [128] used human BMSCs as seed cells and found that BMP-7-functionalized Rada16-1 could promote the differentiation of human BMSCs into nucleus pulposus cells, suggesting that this functional self-assembled polypeptide hydrogel may be a potential treatment for IDD.

These studies indicate that this functional self-assembled polypeptide hydrogel has excellent potential for the regeneration of IVD. The functional self-assembled polypeptide hydrogel has strong mechanical properties and good biocompatibility and can promote the differentiation of nucleus pulpous cells. However, the application of functional self-assembled polypeptide hydrogel requires further study to elucidate the molecular mechanisms of its promotion of IVD regeneration to provide new ideas and methods for the regeneration of IVD.

### 8.4. Applications of Hydrogels Capable of Stem Cell Recruitment in IVD Regeneration

Although stem cell therapy for IDD is a promising therapeutic method, drawbacks include limited sources of stem cells, complex techniques, and high medical costs [129]. As the degenerative disc microenvironment has high osmotic pressure, an acidic pH, low oxygen, and an insufficient supply of nutrients, it is not conducive to stem cell survival [130]. Some biomaterials, especially hydrogels, can effectively overcome this low cell viability environment when mediating the transplantation of stem cells to the diseased site [131]. However, the long-term survival of the transplanted cells remains unknown, especially given the hypoxic, low-nutrient condition within the degenerative IVD [132]. Prior works have proposed the existence of migratory pathways connecting the annulus fibrosus to the nucleus pulposus, which may represent a promising therapeutic option for stem cell therapy in IVD [133]. Chemokine ligand 5 (CCL5) can recruit a large number of cells, including BM-MSCs expressing its specific membrane receptor CCR1/3/5. Frapin et al. [134] developed a pullulan microsphere (PMB) delivery system that sequentially releases CCL5 and growth factors. Endogenous stem cells are first recruited into the degenerated nucleus pulposus via CCL5. Growth factors are then locally released from the PMB to stimulate these migrated cells and promote the synthesis of healthy ECM. Lu et al. [135] constructed a composite hydrogel scaffold by combining a directed acellular cartilage matrix (ACM) with a bone marrow homing peptide- (BMHP-) functionalized self-assembly peptide (SAP). The functional SAP hydrogel promoted the proliferation and differentiation of rabbit MSCs *in vitro*, and *in vivo* application of this hydrogel promoted endogenous stem cell homing and improved cartilage repair.

hMSCs can also migrate to damaged tissues via several growth factors: chemokines [CXCL12/SDF-1(stromal cell-derived factor-1) and MDC (macrophage-derived protein)]. Selecting appropriate vectors and locally increasing the release of cytokines/chemokines can improve the migration hMSCs. Pereira et al. [136] selected SDF-1 chemokines and coated SDF-1 with a hyaluronic acid-poly(N-isopropyl acrylamide) (HAP) hydrogel. The hydrogel can be rapidly cross-linked at temperatures greater than 30° and is biocompatible, making it suitable for the treatment of IDD. Their experiments showed that the HAP hydrogel could recruit hMSCs into the injured disc sites (Figure 5(c)). Importantly, HAP hydrogels also promoted the induction and transduction of the recruited stem cells, thereby promoting nucleus pulposus cell-like differentiation. To prolong the release time of SDF-1 in the hydrogel, Ham et al. [137] co-cross-linked heparin methacrylate with methyl acrylamide chitosan to form a hydrogel. SDF-1 could be released continuously within two weeks because heparin can adsorb chemokines and improve their biologic stability. The recruitment of stem cells with a hydrogel for cell-based therapy is viable. It is expected that more efficient and safe hydrogel biomaterials with improved recruitment function will be developed in the future.

## 9. Summary and Outlook

In this review, we selected some examples to summarize the recent application of hydrogels in the regeneration of the IVD. IDD is caused by multiple factors such as genetics, the environment, and cell senescence. Not only do inflammatory mediators and physical load play an essential role in IDD, but the progressive decrease in nutrient supply and ECM are equally significant influences. The degeneration and regeneration of the IVD is a complex process that involves the ECM of the nucleus pulposus. Hydrogels that are analogs of the ECM provide structural support for the regeneration of nucleus pulposus cells, guide the differentiation of nucleus pulposus cells, promote the production of ECM, and act as a carrier of drugs or stem cells, all of which make them compelling candidate materials for use in IDD and IVD regeneration. More importantly, recently developed multifunctional hydrogels further increase the potential treatment options for IDD, such as by providing a gene-hydrogel microenvironment at the IDD site, which can directly regulate the metabolic balance of the ECM in the nucleus pulposus cells. Furthermore, the responsive hydrogel allows for controllable release at the inflammatory site and delivers drugs on demand. IPN hydrogels achieve biomimetic mechanical strength, thereby supporting and retaining the ECM produced by the nucleus pulposus cells. Hydrogel microspheres are novel drug delivery vectors that are able to be delivered in a minimally invasive fashion via injection with tiny needles. While hydrogels appear to be able to regenerate the diseased IVD, most of the literature remains in animal models so as to permit an assessment of the mechanisms behind hydrogel function. Animal IDD models cannot imitate the natural processes that result in human IDD, and clinical applications are therefore far off.

Future multifunctional hydrogels should possess a bionic mechanical structure, modulate the immune response, and be biodegradable. We present the following recommendations regarding their development:

1. The intervertebral disc is a deep tissue that is adjacent to important nerves and blood vessels. It is therefore an important safety issue to ensure that the hydrogel does not leak during and after implantation. The clinical safety of hydrogels developed in the future must be considered
2. The harsh microenvironment of the degenerative IVD is an important influencing factor for biologic and cellular therapy. Improving the local microenvironment via cellular therapy should be a direction for future research
3. Most drug-carrying hydrogels for the treatment IDD treatment are currently unable to maintain a long-term therapeutic effect and may require repeated injections if used clinically. A hydrogel material that possesses an anti-inflammatory effect may yield an improved therapeutic effect [138]
4. Some patients with low back pain not only have IDD but may also have a neurologic injury. Combining a hydrogel with nerve repair vectors may make it more useful in this field
5. IVD regeneration cannot be separated from its nutritional supply. However, the IVD is an avascular tissue, with a small number of blood vessels and nerves distributed outside the annulus fibrosus. It is therefore important to develop a hydrogel that can provide nutritional support for the regenerating disc
6. The hydrogels that are currently used in the treatment of IDD are currently focused on cell or drug delivery. How to release these vectors sustainably to permit continuous activity still requires further research and exploration
7. The immune microenvironment has been shown to play an essential role in IVD regeneration. Various molecules in the IVD have been shown to inhibit the infiltration of immune cells. When IVD immunity is destroyed, a robust autoimmune response occurs in the human body. How to use hydrogels to regulate the immune system while repairing the IVD should be a focus of future research
8. Hydrogels currently used in IVD regeneration are mainly used in cell and animal experiments, and clinical practice remains far off. Animal models that can better simulate human IDD should be used to better guide the development of new multifunctional hydrogels
9. Hydrogels used for IDD regeneration will improve due to our unremitting efforts and research

## Figures and Tables

**Figure 1:** Applications of hydrogels loaded with traditional drugs/growth factors in IVD regeneration. (a) Composite hydrogel (ASP-Lip@GelMA) for preventing recurrence after partial discectomy [70]. (b) Schematic diagram of Rapa-loaded ROS-responsive hydrogel regulating IVD immune microenvironment and ameliorating tissue repair [72]. (c) Chemical structure of FEFKFEFK (F8) peptide and schematic representation of its self-assembly and gelation pathway. F8 hydrogel was injected on the Petri dish using a 21G needle [80].

**Figure 2:** Gene-hydrogel microenvironment for regeneration of IVDD [88]. (a) The construction of gene-hydrogel microenvironment. (b) The Agomir@PEG was injected into the intervertebral space to construct the gene-hydrogel microenvironment. (c–e) The multifunctions provided by the gene-hydrogel microenvironment, matching the regeneration of IVDD.

**Figure 3:** Preparation and characteristics of PM-reinforced alginate hydrogel [94].

**Figure 4:** (a) Schematic illustration for formation of miRNA/PGPC polyplex micelles [108]. (b) Encapsulation of miRNA/PGPC polyplexes in PEG hydrogels in an injectable manner and molecular mechanism of MMP-2 silence in nucleus pulposus cells for fibrosis inhibition. (c) Injection sites in the IVDs of rabbits.

**Figure 5:** Applications of multifunctional hydrogels in IVD regeneration. (a) Schematic of the process for forming cellularized, fiber-reinforced IPNs by combining MSC-seeded agarose and PEG-DA infiltrated into a 3D woven PCL scaffold [117]. (b) Preparation of APETx2-conjugated GelMA microspheres (GA) and cell-laden GA (GNA), and the injection of GNA in the rat model of IVD degeneration [119]. (c) Schematic representation of the experimental design used for cell migration experiments [136].
